# Effects of Eicosapentaenoic Acid and Docosahexaenoic Acid on Prostate Cancer Cell Migration and Invasion Induced by Tumor-Associated Macrophages

**DOI:** 10.1371/journal.pone.0099630

**Published:** 2014-06-12

**Authors:** Cheng-Chung Li, Yu-Chen Hou, Chiu-Li Yeh, Sung-Ling Yeh

**Affiliations:** 1 School of Nutrition and Health Sciences, College of Public Health and Nutrition, Taipei Medical University, Taipei, Taiwan; 2 Department of Surgery, National Taiwan University, Taipei, Taiwan; 3 Department of Nutrition and Health Sciences, Chinese Culture University, Taipei, Taiwan; Philipps University, Germany

## Abstract

Eicosapentaenoic acid (EPA) and docosahexaenoic acid (DHA) are the major n-3 polyunsaturated fatty acids (PUFAs) in fish oil that decrease the risk of prostate cancer. Tumor-associated macrophages (TAMs) are the main leukocytes of intratumoral infiltration, and increased TAMs correlates with poor prostate cancer prognosis. However, the mechanism of n-3 PUFAs on prostate cancer cell progression induced by TAMs is not well understood. In this study, we investigated the effects of EPA and DHA on modulating of migration and invasion of prostate cancer cells induced by TAMs-like M2-type macrophages. PC-3 prostate cancer cells were pretreated with EPA, DHA, or the peroxisome proliferator-activated receptor (PPAR)-γ antagonist, GW9662, before exposure to conditioned medium (CM). CM was derived from M2-polarized THP-1 macrophages. The migratory and invasive abilities of PC-3 cells were evaluated using a coculture system of M2-type macrophages and PC-3 cells. EPA/DHA administration decreased migration and invasion of PC-3 cells. The PPAR-γ DNA-binding activity and cytosolic inhibitory factor κBα (IκBα) protein expression increased while the nuclear factor (NF)-κB p65 transcriptional activity and nuclear NF-κB p65 protein level decreased in PC-3 cells incubated with CM in the presence of EPA/DHA. Further, EPA/DHA downregulated mRNA expressions of matrix metalloproteinase-9, cyclooxygenase-2, vascular endothelial growth factor, and macrophage colony-stimulating factor. Pretreatment with GW9662 abolished the favorable effects of EPA/DHA on PC-3 cells. These results indicate that EPA/DHA administration reduced migration, invasion and macrophage chemotaxis of PC-3 cells induced by TAM-like M2-type macrophages, which may partly be explained by activation of PPAR-γ and decreased NF-κB p65 transcriptional activity.

## Introduction

Prostate cancer is the most common cancer diagnosed among men in developed countries and is the leading cause of cancer deaths worldwide [1]. Despite improvements in various therapeutic approaches in recent years, therapy for patients with advanced prostate cancer still lacks efficacy. The solid tumor is composed of neoplastic cells and stromal components including fibroblasts, endothelial cells, and migratory hematopoietic cells. Macrophages are the most abundant immune cells in the tumor microenvironment, so-called tumor-associated macrophages (TAMs) [2], [3]. TAMs are mainly M2-type macrophages because they express a series of surface markers such as CD36 and CD163 [4]. Also, TAMs were shown to play crucial roles in survival, proliferation, and metastasis of cancer cells, and higher TAMs infiltration is often correlated with a poor prognosis in many tumors, such as prostate cancer. A clinical study performed by Lissbrant et al. [5] found positive correlations of the density of TAMs with prostate tumor cell proliferation and microvessel density. Moreover, TAMs can facilitate cancer cell migration and invasion by secreting factors, such as growth factors, cytokines, chemotactic factors, and matrix metalloproteinases (MMPs) [6]–[9].

Peroxisome proliferator-activated receptors (PPARs) are nuclear receptors and ligand-activated transcription factors in the steroid superfamily. The PPAR family consists of three different subtypes: PPAR-α, PPAR-β/δ, and PPAR-γ. They heterodimerize with the retinoid X receptor (RXR) and regulate target gene expressions by binding to peroxisome proliferator response elements (PPREs) located in the promoter region [10]. PPAR-γ is primarily expressed in adipose tissues and plays important roles in regulating glucose and lipid metabolism and adipocyte differentiation [11]. It was reported that PPAR-γ activation can modulate inflammatory responses and inhibit the development and progression of a wide range of epithelial-derived human cancer cells, including prostate, breast, and colon cancers [12]–[14]. Additionally, induction of PPAR-γ expression was correlated with inhibition of nuclear factor (NF)-κB activity and decreased expressions of angiogenic proteins in non-small cell lung cancer cells. Those findings suggest that inactivation of NF-κB may be involved in a PPAR-γ-dependent pathway [15].

Eicosapentaenoic acid (EPA) and docosahexaenoic acid (DHA) are the two most common long chain n-3 polyunsaturated fatty acids (PUFAs) in fish oil. Epidemiological data showed that consumption of fish is inversely associated with the incidence of and mortality rates from prostate cancer, especially metastatic cancer [16]–[18]. Serum EPA and DHA levels in patients with prostate cancer were lower than those of patients with benign prostate hyperplasia [19]. Growing evidence has demonstrated that n-3 PUFAs exert antitumor properties. However, little attention has been paid to the relationship between n-3 PUFAs and prostate cancer cell progression induced by TAMs. A previous study showed that EPA inhibits human HT-29 colon cancer cell growth, and this effect was the result of PPAR-γ activation [12]. Further, n-3 PUFAs were shown to induce apoptosis through activation of PPAR-γ in prostate cancer cells [20]. Since n-3 PUFAs have been shown to bind efficiently to the ligand-binding domain of PPAR-γ and activate PPAR response element-reporter assays in various cell lines [12], [21], we hypothesized that EPA and DHA administration suppress the progressive properties of prostate cancer via activation of PPAR-γ involved pathway. Thus, we used PC-3 cells treated with conditioned medium (CM) from M2-type macrophages or in a non-contact system to determine the effects and possible mechanisms of EPA and DHA on prostate cancer cell migration and invasion induced by TAMs.

## Materials and Methods

### Cell lines and culture conditions

Prostate PC-3 cancer cells and human THP-1 monocytic cells were obtained from American Type Culture Collection (Manassas, VA, USA). Cells were maintained in RPMI 1640 medium (Invitrogen, Carlsbad, CA, USA) containing 10% fetal bovine serum (FBS), 1% penicillin-streptomycin (10 ng/mL penicillin and 10 U/mL streptomycin), and 2.5 mM glutamine at 37°C in a humidified 5% CO_2_ incubator.

### Preparation of fatty acid-bovine serum albumin (BSA) complexes

EPA, DHA, and BSA were purchased from Sigma (St. Louis, MO, USA). Fatty acid-BSA complexes were prepared as 10 mmol/L stocks with a ratio of fatty acids to BSA of 4∶1 and were solubilized by a sonicator in a cool water bath for 60 min. Fatty acid-BSA stocks were stored at −20°C under argon until ready for use [22].

### Cell viability assay

The viability of PC-3 cells was determined by an Alamar blue assay (Invitrogen). PC-3 cells were seeded into 96-well plates (1000 cells/well) overnight, and then treated with different doses of EPA or DHA (0∼400 µM). BSA vehicle was used as a control (C). After 20 h of treatment, cells were incubated in medium containing 10% Alamar blue dye at 37°C for 4 h, and the colorimetric change was measured with a microplate reader at 570 and 600 nm.

### CM preparations and treatments

Macrophage differentiation was performed according to previously established protocols [23]. THP-1 cells (5×10^6^) were seeded in 75-cm^2^ tissue culture flasks and cultured with 320 nM phorbol 12-myristate 13-acetate (PMA; Sigma) for 4 h. For M2-type macrophage differentiation, THP-1 cells were treated with 320 nM PMA, 20 ng/mL interleukin (IL)-4, and 20 ng/mL IL-13 (PeproTech, Rocky Hill, NJ, USA) for another 20 h. To generate M1-type macrophages, THP-1 cells were treated with 320 nM PMA for 4 h, and then treated with 320 nM PMA, 20 ng/mL interferon (IFN)-γ (PeproTech), and 100 ng/mL lipopolysaccharide (LPS) from *Escherichia coli* serotype 0111:B4 (Sigma) for 20 h. After stimulation, cells were washed with phosphate-buffered saline (PBS) twice and cultured with fresh medium for 24 h, and then CM was collected.

PC-3 prostate cancer cells were seeded at 5×10^5^ in 6-well plates 1 day prior to treatment. To treat cells, cells were placed in medium containing different concentrations of EPA, DHA (0, 25, and 50 µM) or 10 µM GW9662 for 24 h, and then cells were treated with CM containing the same concentration of fatty acids for another 24 h. PC-3 cells were harvested for further analysis.

### Migration and invasion assays

The migratory and invasive abilities of PC-3 cells (2×10^4^ for the migration assay and 10^5^ cells for the invasion assay) were respectively determined using 24-well plates with Millicell Culture Plate Inserts (8-μm pore size; Millipore, Billerica, MA, USA) for 12 h and Matrigel-coated (BD Biosciences, Bedford, MA, USA) inserts for 24 h. Briefly, PC-3 cells were added to the upper compartments in RPMI 1640 supplemented with 10% FBS, and THP-1 cells (10^5^) were differentiated into M2-type macrophages in the lower chambers. After PC-3 cells had attached, medium from the upper and lower chamber were replaced with serum-free RPMI 1640 containing different concentrations of EPA, DHA, or GW9662 (10 µM). Then, cells on the upper insert surface of the membrane were removed with cotton swabs after incubation. After fixation with 4% paraformaldehyde, migrating and invasive cells were stained with 0.5% crystal violet in 2% methanol. Membranes were washed three times with PBS, and the dye was eluted with 30% acetic acid. The absorbance was read at 595 nm with a microplate reader. At least three independent experiments were performed for each assay.

### DNA-binding activities of PPAR-γ and NF-κB p65

Nuclear extracts from cells were harvested using the NE-PER Cytoplasmic and Nuclear Protein extraction kit (Pierce Biotechnology, Rockford, IL, USA) according to the manufacturer's instructions. The DNA-binding activity of PPAR-γ was assayed using an enzyme-linked immunosorbent assay (ELISA)-based Trans-AM Transcription Factor Assay PPAR-γ Kit (Active Motif, Carlsbad, CA, USA). An oligonucleotide that contained a peroxisome proliferator response element (PPRE) (5′-AACTAGGTCAAAGGTCA-3′) was coated onto wells of the microtiter strips provided. PPAR contained in the nuclear extract specially binds to the PPRE. The primary PPAR-γ antibody recognizes an assessable epitope on the PPAR-γ protein upon DNA binding and then a secondary antibody conjugated to horseradish peroxidase (HRP) was added. The absorbance was read using a spectrophotometer at 450 nm.

To quantify the DNA-binding activity of NF-κB p65, 5 µg of the nuclear extract was measured using an ELISA-based Trans-AM Transcription Factor Assay NF-κB p65 Kit (Active Motif). The wells of the ELISA kits were immobilized with an oligonucleotide that contained the NF-κB p65 consensus site (5′-GGGACTTTCC-3′). According to the manufacturer's instructions, 10 µg of the nuclear extract was added to each well, and then incubated with a specific primary antibody used to detect NF-κB that recognizes an epitope on p65 that is accessible only when NF-κB is activated and bound to its target DNA. After incubation with an HRP-conjugated secondary antibody, the colorimetric reaction was quantified using spectrophotometry at 450 nm.

### Protein extraction and Western blot analysis

Cells were washed with ice-cold PBS and scraped in lysis buffer (50 mM Tris at pH 7.4, 1% sodium dodecylsulfate (SDS), 1% Nonidet P-40, 0.5% Na-deoxycholate, 150 mM NaCl, 1 mM EDTA, and 50 mM NaF) containing a protease inhibitor cocktail (Complete, Roche Diagnostics, Mannheim, Germany) to prepare whole-cell lysates. To collect the nuclear and cytoplasmic extracts, cells were harvested using the NE-PER Cytoplasmic and Nuclear Protein extraction kit (Pierce Biotechnology) according to the manufacturer's instructions. Protein concentrations of the supernatant were determined with a Bradford Protein Assay Reagent kit (Bio-Rad, Richmond, CA, USA). Proteins were electrophoresed onto 4%∼12% SDS-polyacrylamide gel electrophoresis (PAGE), and transferred onto polyvinylidene difluoride membranes in a wet-transfer apparatus. Membranes were blocked with 5% nonfat milk in TBS-Tween (TBS-T) for 1 h and then incubated with a specific primary antibody overnight at 4°C. Membranes were washed three times with TBS-T and incubated with HRP-conjugated secondary antibodies for 1 h, and blots were developed with enhanced chemiluminescence reagents (PerkinElmer Life Sciences, Waltham, MA, USA) and exposed to x-ray film. Relative intensities were measured to quantify protein levels using Image-Pro Plus software (Media Cybernetics, Bethesda, MD, USA). All blots were quantified and normalized against an internal control to adjust for the amount of proteins loaded.

### RNA extraction and real-time polymerase chain reaction (PCR) analysis

Total RNA from cells was extracted using the Trizol reagent (Invitrogen). Concentrations of RNA were determined and quantified by measuring the absorbance at 260 and 280 nm on a spectrophotometer. Complementary (c)DNA was synthesized from total RNA using a cDNA synthesis kit (Fermentas, Glen Burnie, MD, USA). A real-time PCR analysis was performed using the ABI 7300 Real-Time PCR System (Applied Biosystems, Foster City, CA, USA) with Maxima SYBR Green qPCR Master Mix (Thermo Scientific, Foster City, CA, USA) to determine each mRNA expression. Primers for CD36, CD163, PPAR-γ, MMP-9, tissue inhibitor of metalloproteinase (TIMP)-1, VEGF, cyclooxygenase (COX)-2, macrophage colony-stimulating factor (M-CSF), and β-actin are listed in Table 1. Reactions were carried out in a total volume of 25 µl containing 1× Maxima SYBR Green qPCR Master Mix, 400 nM of each primer, and 100 ng of cDNA. The cycling conditions were as follows: 50°C for 2 min and 95°C for 10 min, followed by 40 cycles of 95°C for 15 s and 60°C for 1 min. mRNA expressions were quantified in duplicate. Data were calculated by the equation 2^−ΔΔCT^ and presented as the multiples of change in gene expression normalized to β-actin.

**Table 1:** Sequences of oligonucleotide primers used in the PCR amplification.

Gene	Forward primer	Reverse primer	Accession number
CD36	5′-AGCCTCATTTCCACCTTTTG-3′	5′-TGGGTTTTCAACTGGAGAGG-3′	XM_005630893
CD163	5′-TGTGGCCTGCATAGAGAGTG-3′	5′-TTCCCCAAAATGAGCAGAAC-3′	XM_005253529
PPAR-γ	5′-GACCACTCCCACTCCTTTGA-3′	5′-AGGCTCCACTTTGATTGCAC-3′	NM_138711
M-CSF	5′-ATGCGCTTCAGAGATAACACC-3′	5′-TTCTTGACCTTCTCCAGCAAC-3′	NM_172211
COX-2	5′-CCCTTGGGTGTCAAAGGTAA-3′	5′-GCCCTCGCTTATGATCTGTC-3′	XM_001107538.2
MMP-9	5′-GGGACGCAGACATCGTCATC-3′	5′-TCGTCATCGTCGAAATGGGC-3′	NM_004994
TIMP-1	5′-CTTCTGCAATTCCGACCTCGT-3′	5′-CCCTAAGGCTTGGAACCCTTT-3′	XM_005272645
β-actin	5′- CATGTACGTTGCTATCCAGGC -3′	5′- CTCCTTAATGTCACGCACGAT-3′	NM_001101

### Enzyme-linked immunosorbent assay (ELISA)

Levels of tumor necrosis factor (TNF)-α, IL-1β, and IL-6, transforming growth factor (TGF)-β, monocyte chemoattractant protein (MCP)-1, and IL-8 were measured using ELISA kits (eBioscience San Diego, CA, USA). The surfaces of the microplates were coated with an MCP-1 or IL-8 human monoclonal antibody. Prostaglandin (PG)E2 concentrations were assayed by a competitive sandwich ELISA kit (R&D Systems, Minneapolis, MN, USA). Procedures followed the manufacturer's instructions. The PGE2 ELISA had an intraplate coefficient of variation (CV) range of 5.9%∼10.3% with a mean assay detection limit of 27.5 pg/mL.

### Statistical analysis

All data are expressed as the mean ± standard deviation (SD). All statistical analyses were performed with GraphPad Prism 5 software. Differences among groups were analyzed by an analysis of variance (ANOVA) followed by Tukey's post-hoc test. A *p* value of <0.05 was considered significantly different.

## Results

### Expression of surface markers and cytokines levels in CM from PMA-treated THP-1 macrophages

To determine whether TAMs-like M2-type macrophages were successfully produced, THP-1 cells were co-treated with PMA and TH2 cytokines (IL-4 and IL-13). The result showed that, compared to PMA-treated only and M1-polarized THP-1 macrophages, M2-type macrophages produced significantly higher mRNA expressions of M2 macrophage markers CD36 and CD163 (Figure 1). Since M2-type macrophages produce relatively lower levels of TNF-α, IL-1β, and IL-6 and higher levels of TGF-β compared to M1-type macrophages. The levels of these cytokines in CM can be used to evaluate the polarization of THP-1 macrophage. We found that CM from the PMA and M2 groups had significantly lower TNF-α, IL-1β, and IL-6 levels than the M1 group. In addition, the CM from the M2 groups had significantly higher TGF-β levels than that in the PMA and M1 groups (Figure 2).

**Figure 1:** Expression of markers for M2-type macrophages in phorbol 12-myristate 13-acetate (PMA)-treated THP-1 macrophages. THP-1 cells treated with 320 nM PMA for 4 h, and then cultured with PMA plus 20 ng/mL interleukin (IL)-4 and 20 ng/mL IL-13 for another 20 h had significantly higher mRNA expressions of CD36 and CD163 (both markers of M2 macrophages) compared to those of M1-polarized THP-1 macrophages. mRNA expression was analyzed by a real-time PCR. Multiples of mRNA changes were quantitated by the comparative CT method. All data are presented as the mean ± SD, *n* = 6. Means with different letters significantly differ (*p*<0.05).

**Figure 2:** Cytokine profiles in conditioned medium (CM) from PMA-treated THP-1 macrophages. CM from PMA-treated THP-1 macrophages and M2-polarized THP-1 macrophages both had significantly lower levels of tumor necrosis factor (TNF)-α (A), interleukin(IL)-1β (B), and IL-6 (C), and a higher level of transforming growth factor (TGF)-β (D) compared to those of M1-polarized THP-1 macrophages. TNF-α, IL-1β, IL-6, and TGF-β were measured by ELISAs. Data are presented as the mean ± SD, *n* = 6. Means with different letters significantly differ (*p*<0.05).

### PC-3 prostate cancer cell viability

The effects of EPA and DHA on PC-3 cell viability were determined by an Alamar blue assay, and results are shown in Figure 3. The viability of PC-3 cells was significantly reduced upon a 24-h exposure to EPA and DHA in a concentration-dependent manner above 150 and 100 µM, respectively.

**Figure 3:** Effects of different eicosapentaenoic acid (EPA) and docosahexaenoic acid (DHA) doses on PC-3 prostate cancer cell viability. PC-3 cells were incubated with EPA (A) and DHA (B) for 24 h followed by an Alamar blue assay performed in quadruplicate. Data are presented as the mean ± SD, *n* = 6. * Significantly differs from the control (*p*<0.05).

### Migratory and invasive abilities in PC-3 prostate cancer cells cocultured with M2-type macrophages

To determine if EPA and DHA are involved in M2-type macrophages-induced prostate cancer cells migration and invasion, PC-3 cells were cocultured with M2-type macrophages in a noncontact apparatus. Migratory and invasive abilities were upregulated in PC-3 cells cocultured with M2-type macrophages. EPA and DHA both significantly reduced the migratory and invasive abilities of PC-3 cells cocultured with M2-type macrophages in dose-dependent fashions. Approximately 80% of the reduction in the migratory and invasive cells was reversed in the presence of GW9662, supporting PPAR-γ activation being involved in inhibiting the migratory and invasive abilities of PC-3 cells cocultured with M2-type macrophages (Figure 4, 5).

**Figure 4:** Effects of EPA and DHA on PC-3 prostate cancer cell M2-type macrophage-induced migration. PC-3 cells were seeded in the upper chambers and cocultured with M2-polarized THP-1 macrophages in the presence of 50 µM EPA, DHA, or GW9662 (10 µM) for 24 h. Invaded cells were fixed in 4% paraformaldehyde and stained with 0.5% crystal violet. Membranes were washed and the dye was eluted with a violet extraction solution (50% ethanol, 0.1% acetic acid, and 49.9% ddH_2_O). The absorbance was measured at 595 nm using a microtiter plate reader. Data are presented as the mean ± SD, *n* = 3. Means with different letters significantly differ (*p*<0.05).

**Figure 5:** Effects of EPA and DHA on PC-3 prostate cancer cell M2-type macrophage-induced invasion. For the invasion assay, PC-3 cells were seeded in the upper chambers coated with Matrigel and cocultured with M2-polarized THP-1 macrophages in the presence of 50 µM EPA, DHA, or GW9662 (10 µM) for 24 h. Invaded cells were fixed in 4% paraformaldehyde and stained with 0.5% crystal violet. Membranes were washed, and the dye was eluted with a violet extraction solution (50% ethanol, 0.1% acetic acid, and 49.9% ddH_2_O). The absorbance was measured at 595 nm using a microtiter plate reader. Data are presented as the mean ± SD, *n* = 3. Means with different letters significantly differ (*p*<0.05).

### EPA and DHA upregulated DNA-binding activity, and protein and mRNA expressions of PPAR-γ in PC-3 cells incubated with CM from M2-type macrophages

EPA and DHA both are ligands of PPAR-γ. To determine whether EPA and DHA reduced migratory and invasive abilities of PC-3 cells through activating PPAR-γ, we analyzed the PPAR-γ DNA-binding activity, mRNA and protein expressions in PC-3 cells cultured with CM from M2-type macrophages. PPAR-γ DNA-binding activity was suppressed in PC-3 cells incubated with CM from M2-type macrophages. Treatment with EPA and DHA both significantly increased the DNA-binding activity, and mRNA and protein expressions of PPAR-γ in PC-3 cells compared to PC-3 cells along with CM from M2-type macrophages. GW9662 partially blocked PPAR-γ activation in PC-3 cells (Figure 6).

**Figure 6:** DNA-binding activity, and protein and mRNA expressions of peroxisome proliferator-activated receptor (PPAR)-γ in PC-3 cells incubated with CM from M2-type macrophages in the presence of EPA, DHA, or GW9662. The PPAR-γ-binding activity was analyzed by a transcription factor ELISA (A). PPAR-γ protein levels were determined by Western blotting (B). Equal protein loading was confirmed using β-actin. mRNA expression of PPAR-γ was analyzed by a real-time PCR (C). mRNA changes were quantitated by the comparative CT method. Data are presented as the mean ± SD, *n* = 3, and means with different letters significantly differ (*p*<0.05).

### EPA and DHA reduced NF-κB activation in PC-3 cells incubated with CM from M2-type macrophages

PPAR-γ activation may decrease DNA-binding activity of NF-κB p65. As shown in Figure 7A, NF-κB p65 DNA-binding activity was upregulated in the absence of EPA/DHA, and declined with administration of EPA/DHA. Treatment with EPA and DHA both significantly decreased nuclear NF-κB p65 protein expression and increased cytosolic IκBα protein expression in dose-dependent manners. Administration of GW9662 significantly reversed the EPA- or DHA-mediated inactivation of NF-κB in PC-3 cells cultured with CM from M2-type macrophages (Figure 7B, C).

**Figure 7:** Nuclear factor (NF)-κB DNA-binding activity, protein expression of the nuclear NF-κB p65 subunit and cytosolic inhibitory factor κBα (IκBα) in PC-3 cells incubated with CM from M2-type macrophages in the presence of EPA, DHA, or GW9662. The NF-κB DNA-binding activity was analyzed by a transcription factor ELISA (A). Protein levels of the IκBα subunit (B) and NF-κB p65 (C) were determined by Western blotting. Equal loading of proteins is illustrated by tubulin bands in the cytosolic fraction. Histone H1 expression is shown as an internal control in nuclear extracts. Data are presented as the mean ± SD, *n* = 3, and means with different letters significantly differ (*p*<0.05).

### Angiogenic-related factor expressions in PC-3 cells cultured with CM from M2-type macrophages

TAMs may enhance the angiogenic potential of cancer cells. We analyzed angiogenic-related factors in PC-3 cells incubated with CM from M2-type macrophages. TAMs induction of mRNA expressions of MMP-9, VEGF, COX-2, and higher levels of PGE2 and IL-8 were found in PC-3 cells cultured with CM from M2-type macrophages (Figure 8). These angiogenic-related factors were downregulated in the presence of EPA/DHA. Treatment with EPA/DHA effectively upregulated mRNA expression of TIMP-1. Regulation of angiogenic-related factors expressions by EPA/DHA in PC-3 cells cultured with CM from M2-type macrophages was abolished by cotreatment with GW9662.

**Figure 8:** mRNA expressions of matrix metalloproteinase (MMP)-9 (A), tissue inhibitor of metalloproteinase (TIMP)-1 (B), vascular endothelial growth factor (VEGF) (C), and cyclooxygenase (COX)-2 (D) and levels of prostaglandin (PG)E2 (E) and interleukin (IL)-8 (F) in PC-3 cells incubated with CM from M2-type macrophages in the presence of EPA, DHA, or GW9662. mRNA expressions were analyzed by a real-time PCR. mRNA changes were quantitated by the comparative CT method. Levels of PGE2 and IL-8 were analyzed by ELISAs. Data are presented as the mean ± SD, *n* = 6, and means with different letters significantly differ (*p*<0.05).

### Gene expression of M-CSF and MCP-1 level in PC-3 cells cultured with CM from M2-type macrophages

Growth factors and chemokines are important for regulating macrophage recruitment to the tumor sites. Our results showed that gene expression of M-CSF and concentrations of MCP-1 in PC-3 cells cultured with CM from M2-type macrophages were upregulated (Figure 9). Gene expression of M-CSF and production of MCP-1 were reduced by EPA/DHA administration. However, treatment with GW9662 was able to reverse the EPA/DHA-mediated downregulation of M-CSF and MCP-1.

**Figure 9:** Production of monocyte chemoattractant protein (MCP)-1 (A) and mRNA expression of macrophage colony-stimulating factor (M-CSF) (B) in PC-3 cells incubated with CM from M2-type macrophages in the presence of EPA, DHA, or GW9662. The MCP-1 level was analyzed by an ELISA. M-CSF was analyzed by a real-time PCR. mRNA changes were quantitated by the comparative CT method. Data are presented as the mean ± SD, *n* = 6, and means with different letters significantly differ (*p*<0.05).

## Discussion

Previous studies reported that n-3 PUFAs inhibit prostate cancer cell growth by inducing apoptosis. In this study, we investigated the potential mechanisms of n-3 PUFAs in modulating of PC-3 cells cultured with CM from M2-type macrophages. Our study is the first to report that compared to PC-3 cells cultured with CM from M2-type macrophages, administration of EPA/DHA reduced migratory and invasive abilities through enhancing PPAR-γ DNA-binding activity, downregulating activation of NF-κB, and repressing the expression of NF-κB-targeted genes.

Macrophages have multiple subtypes and can be polarized by distinct stimuli. M1-type macrophages have anti-tumor properties and are characterized by production high level of TNF-α, IL-1β, and IL-6. M2-type macrophages show tumor-growth promoting properties and express higher immunosuppressive cytokines, such as TGF-β. These cytokines markers were used to define M1- and M2-type macrophages polarization. We observed that PMA-, IL-4-, and IL-13-treated THP-1 cells showed M2-type macrophage surface markers of CD36 and CD163 and M2-type macrophages cytokine profiles (lower concentrations of TNF-α, IL-1β, and IL-6, and a higher concentration of TGF-β). Within the tumor microenvironment, TAMs primarily exhibit an M2-type macrophages functional profile, and this preferred polarization is due to stimulation by TH2 cytokines [24], [25]. TH2-derived cytokines, IL-4 and IL-13, induce M2 polarization of TAMs leading to tumor promotion and development [26], [27]. Macrophage recruitment and differentiation of M2-type macrophages are regulated by growth factors such as M-CSF and chemokines including MCP-1 [28]. Overexpression of M-CSF and MCP-1 in several types of cancers, including prostate cancer, increases macrophage recruitment and tumor progression, and accelerates the rate of metastasis [29]–[32]. M-CSF binding to colony-stimulating factor-1 receptor can stimulate macrophage differentiation and predict caner metastasis. A slower rate of tumor progression and inhibition of metastasis were found in breast cancer after genetic ablation of M-CSF [33]. Also, reductions in growth and macrophage recruitment were found in PC-3 cells after MCP-1 antibody neutralization [30]. Results of this study showed that EPA/DHA may decrease the ability of macrophage recruitment in PC-3 cells cultured with CM from M2-type macrophages by downregulating M-CSF and MCP-1.

A previous study revealed that M2-polarized THP-1 macrophages can induce invasion and angiogenesis of human basal carcinoma cells [23]. We also found that TAM-like M2-type macrophages elevated the migration and invasion of PC-3 prostate cancer cells. Furthermore, administration of EPA/DHA suppressed the migratory and invasive properties of PC-3 cells induced by TAM-like M2-type macrophages, whereas ∼80% of this effect was blocked by co-treatment with GW9662, a PPAR-γ-specific antagonist. Evidence suggests that the endogenous PPAR-γ ligand, 15-deoxy-Δ^12,14^-prostaglandin J_2_ (15d-PGJ_2_) suppressed proliferation of and androgen signaling by prostate cancer cells [34], [35]. Also, treatment with 15d-PGJ_2_ and the synthetic ligand, pioglitazone, was reported to inhibit the proliferation and invasion ability of human colon cancer cells [36]. PPAR-γ is expressed in the human prostate epithelium. Although prostate carcinomas was found to overexpress PPAR-γ [13], activation of PPAR-γ was shown to inhibit the growth of prostate cancer cells and cancer progression [37].

Transcriptional activity of NF-κB is mainly modulated by phosphorylation and nuclear translocation of NF-κB p65 [38]–[40]. Abnormal NF-κB activation was identified in cancer cells, which promoted invasion and migration by increasing expressions of MMPs and vascular endothelial growth factor (VEGF) in prostate cancer PC-3 cells [41]. Previous studies indicated that PPAR-γ competes with NF-κB to bind co-activators of the steroid receptor co-activator (SRC)-1 or cAMP-response element-binding (CREB) protein which inhibits NF-κB-mediated gene expression [42]. Also, PPAR-γ activation may induce the synthesis of IκBα, which directly binds to p65 containing NF-κB dimers in the cytoplasm and inhibits the nuclear translocation of NF-κB [43], [44]. In the present study, we found that EPA and DHA increased cytosolic IκBα expression in PC-3 cells cultured in CM. These data suggest that EPA and DHA modulate the migratory and invasive properties of PC-3 cells induced by M2-type macrophages in part by enhancing the PPAR-γ DNA-binding activity and decreasing the NF-κB p65 transcriptional activity. Recently, n-3 PUFAs were reported to activate G protein-coupled receptor (GPR) 120 and inhibit NF-κB activity that may consequently attenuate proinflammatory cytokines secretion and modulate adipose tissue inflammation [45]. We did not consider the inhibitory effect of NF-kB by n-3 PUFA via GPR120 because the beneficial effect of n-3 PUFA was almost abolished by co-treatment with GW9662. Although the interaction between n-3PUFA and GPR120 cannot be excluded, our study can prove, at least, that activation of PPAR-γ is one of the mechanisms responsible for reducing migratory and invasive abilities of prostate cancer cells induced by TAMs.

Downregulation of NF-κB downstream targets such as MMP-9, COX-2, VEGF, and IL-8 plays important roles in inhibiting cancer cell migration, invasion, and metastasis [46], [47]. MMP-9 is one of the most crucial MMPs that degrade the extracellular matrix (ECM) and further stimulate other growth factors to facilitate the migration and invasion of cancer cells [48]. The main natural inhibitor of MMP-9 is TIMP-1. The C-terminal domain of TIMP-1 binds to the hemopexin-like domain of MMP-9 [49]. The MMP-9/TIMP-1 ratio may represent the proteolytic ability of numerous cancer cells [50], [51]. IL-8 and VEGF are two multifunctional cytokines and were demonstrated to correlate with the malignant potential. VEGF is one of the most important factors for neovascularization in cancer cells. Previous study showed that downregulation of VEGF expression can suppress prostate tumor growth and progression [52]. IL-8 signaling can promote angiogenic responses in endothelial cells and increase the growth rate and invasive ability of cancer cells by inducing additional growth factor secretion from TAMs [53]. Serum IL-8 is higher in prostate cancer patients with bone metastasis than in localized prostate cancer [54]. It is widely reported that COX-2 and its product, PGE2, were correlated with progression of a number of types of cancers, such as prostate cancer [55], [56]. Results of our study consistent with the previous reports that gene expressions of MMP-9, VEGF, and COX-2 and levels of IL-8 and PGE2 in PC-3 cells cultured with CM from M2-type macrophages were upregulated. A study conducted by Kobayashi et al. [57] indicated that dietary n-3 fatty acids alter prostate tumor membrane n-6/n-3 ratios, thus decreasing COX-2 protein expression and production of PGE2 which are implicated in reducing prostate cancer invasion and metastasis. Our findings also showed that EPA/DHA administration reduced expressions of these parameters in PC-3 cells cultured with CM that may consequently lead to inhibition of cell migration and invasion. The dosage of EPA/DHA used in this study was comparable to plasma n-3 levels with high fish consumption subjects [58]. Although this in vitro study cannot accurately reflect the integrative nature in the human body, it provides basic information and implies an additional rationale for evaluating EPA/DHA supplementation in patients with prostate cancer.

In summary, the present study showed that TAM-like M2-type macrophages enhanced the migration and invasion of PC-3 prostate cancer cells. EPA and DHA administration both suppressed the migratory and invasive properties of PC-3 cells induced by TAM-like M2-type macrophages, which may partly be explained by activation of PPAR-γ and downregulation of NF-κB transcriptional activity. Also, treatment with EPA and DHA decreased expressions of NF-κB-targeted genes that may reduce the chemotactic ability of PC-3 cells for macrophages.
